The article "Knockdown of miR-372-3p Inhibits the Development of Diabetic Cardiomyopathy by Accelerating Angiogenesis via Activating the PI3K/AKT/mTOR/HIF-1α Signaling Pathway and Suppressing Oxidative Stress" was retracted in 2023. Reasons: unreliable results or conclusions; concerns about the data; concerns about the peer review; concerns about the citations.

# Knockdown of miR-372-3p Inhibits the Development of Diabetic Cardiomyopathy by Accelerating Angiogenesis via Activating the PI3K/AKT/mTOR/HIF-1*α* Signaling Pathway and Suppressing Oxidative Stress

**DOI:** 10.1155/2022/4342755

**Published:** 2022-09-16

**Authors:** Zhimin Han, Danyang Zhao, Mengfan Han, Rongjin Zhang, Yongmei Hao

**Affiliations:** ^1^Academic Affairs Office, The Second Hospital of Hebei Medical University, Shijiazhuang 050000, China; ^2^Department of Endocrinology, The Second Hospital of Hebei Medical University, Shijiazhuang 050000, China; ^3^Department of Psychosomatic Medicine, The Second Hospital of Hebei Medical University, Shijiazhuang 050000, China

## Abstract

**Background:**

DCM is the most common and malignant complication of diabetes. It is characterized by myocardial dilatation, hypertrophy, fibrosis, ventricular remodeling, and contractile dysfunction. Although many studies have demonstrated the function of miRNAs in the progression of DCM, but the specific role of miR-372-3p in DCM remains unknown.

**Methods:**

C57/BL6J mice were used to construct mouse models of DCM by intraperitoneal injection of STZ (50 mg/kg/d) for 5 consecutive days. Then the mice were randomly divided into model group (intramyocardial injection of empty lentivirus) and miR-372-3p KD group (intramyocardial injection of miR-372-3p KD lentivirus at 10^9^/mouse). Besides, the control group (injection of 0.9% normal saline) was also set up. LY294002, a PI3K inhibitor, was employed in the current study. Western blotting, immunofluorescence staining, quantitative ultrasound method, Masson's trichrome staining, and bioinformatics analysis were performed.

**Results:**

It was found that miR-372-3p KD significantly improved left ventricular dysfunction and cardiac hypertrophy in DCM mice. Furthermore, it also improved myocardial interstitial fibrosis and remodeling in DCM mice. Immunofluorescence staining and RT-qPCR revealed that miR-372-3p KD might accelerate cardiac remodeling by increasing angiogenesis in DCM mice. Western blotting results revealed that miR-372-3p was an upstream target of the PI3K/AKT-mTOR and HIF-1*α* signals, as well as NOX2, NOX4, which were responsible for angiogenesis in DCM mice. Besides, the *in vitro* experiment showed that LY294002 markedly diminished the increased expression levels of p-PI3K, AKT, p-mTOR, p-P70S6K, HIF-1*α*, NOX2, and NOX4 in the model group and the miR-372-3p KD group, suggesting that PI3K signaling pathway and oxidative stress are involved in miR-372-3p KD-induced angiogenesis in HG-stimulated C166 cells.

**Conclusions:**

MiR-372-3p KD inhibits the development of DCM *via* activating the PI3K/AKT/mTOR/HIF-1*α* signaling pathway or suppressing oxidative stress. This offers an applicable biomarker for DCM treatment.

## 1. Introduction

DCM, a chronic complication of diabetes mellitus, brings a heavy burden to the patient's family and the society [1, 2]. Some cardiac anomalies are detected in DCM patients, including myocardial dilatation, hypertrophy, fibrosis, ventricular remodeling, contractile dysfunction, and vascular system disorders, which can lead to heart failure and increase the death rate [3–5]. So far, there are no effective therapeutic regimens to block the pathological changes associated with DCM. Therefore, it is urgent to elucidate the pathogenesis of DCM and determine its therapeutic hallmark.

As reported previously, VEGFs can accelerate angiogenesis, improve myocardial contractility, diminish cardiac hypertrophy effectively constrain ventricular renovation, and improve cardiac functions [6–8]. Angiogenesis plays a crucial role in tissue progression, and homeostasis and impaired angiogenesis are closely related to several diseases, including DCM [9, 10].

The PI3K is a critical progrowth cell signal implicated in numerous pathological and physiological processes, which can phosphorylate serine/threonine kinase AKT [11–13]. Additionally, numerous studies have demonstrated that mTOR is a downstream protein complex (mTORC1 and mTORC2) involved in the PI3K/AKT pathway and regulates cell proliferation, protein synthesis, and angiogenesis [14–16]. Furthermore, P70S6K is activated by mTOR and serves as a critical regulator in the progression and functions of blood vessels [17, 18]. Numerous previous studies have highlighted that the PI3K/AKT/mTOR/p70S6K signaling pathway plays a vital role in the development of neovascularization [19–21]. HIF-1*α* is another crucial downstream protein of mTOR, which plays a vital role in cell proliferation and angiogenesis [22, 23]. The long-term exposure to hyperglycemia in the heart could produce the amount of oxidative stress induce in the overproduction of ROS, which is derived from NOX, especially NOX2 and NOX4 which are important sources of O^2−^ and H_2_O_2_; all of these responses result into a serious deteriorating consequence, such as mitochondrial dysfunction, advanced glycation end products, calcium overload, lipotoxicity, and inflammation, all eventually promote the progression of DCM, and moreover, the oxidative stress is also toxic for systolic and endothelial dysfunction and cardiac cell death and necrosis; thereby the reduction of oxidative stress is an attractive target for cure of cardiac diseases. PI3K/AKT signaling pathway has been reported to suppress inflammation and mediate oxidative stress, thereby any interfering factor with anti-inflammatory or antioxidant features may be beneficial for DCM [24–26].

miRNAs are small, noncoding RNAs that act as crucial posttranscriptional regulators of gene expression by binding to the UTRs of large target mRNAs [27, 28]. As an essential member of the miRNA family, miR-372-3p has drawn our attention; it is a highly conserved miRNA among humans and animals [29, 30]. However, the specific role of miR-372-3p in DCM has rarely been reported. Therefore, miR-372-3p expression came into the spotlight of this study. We conducted a series of *in vivo* and *in vitro* experiments to determine the role of miR-372-3p in DCM.

## 2. Materials and Methods

### 2.1. Mice

In this study, 6-8-week-old C57BL/6 J mice (Skbex Biotechnology) were used to establish mouse models of diabetes mellitus by intraperitoneal injection of STZ (50 mg/kg/d) for 5 consecutive days. Then the fasting blood glucose (>16.7 mmol/L) was extracted from the tail vein for later use. The mice were randomly divided into model group (intramyocardial injection of empty lentivirus) and miR-372-3p KD group (intramyocardial injection of miR-372-3p KD lentivirus at 10^9^/mouse). Besides, control group (injection of 0.9% normal saline) was also set up. All the mice were kept in SPF-level animal laboratory with a 12 : 12-h light-dark cycle at 24-26°C, where they were bred adaptively for one week prior to the experiment.

### 2.2. Mouse Heart Ultrasound

db/db mice were anesthetized with isoflurane after chest depilation. The LVIDd and LVIDs of mice in each group were detected by high-resolution small animal ultrasound imaging system. In addition, the LVFS and EF were calculated. Three consecutive cardiac cycles were detected, and the average value was taken.

### 2.3. Masson's Trichrome Staining

The tissues were routinely dehydrated and embedded. Then the obtained tissues were cut into 4-*μ*m-thick sections and conventionally dewaxed to water. Next, the sections were mordanted overnight at room temperature, stained with celestine blue staining solution for 2-3 min, with Mayer's hematoxylin staining solution for 2-3 min and with acid ethanol differentiation solution for 2-3 min. After that, the samples were washed by water for 10 min and stained with fuchsin staining solution for 10 min, with molybdophosphoric acid solution for 10 min, and with aniline blue dye for 5 min. After aniline blue solution was rinsed off with weak acid solution, weak acid solution was added again to cover the slices for 2 min. Finally, the sections were sealed using neutral gum. The blue stained parts were the fibrotic areas, and the ratio of these part vs. total myocardial areas was used to calculate the area of fibrosis.

### 2.4. *α*-SMA, CD31, and Collagen-III Immunofluorescence Staining

The paraffin-embedded tissues were cut into 4*-μ*m-thick sections. After routine dewaxing and dehydration, the antigen was restored at high temperature. Then the sections were incubated with 3% H_2_O_2_ for 30 mi and with 3% goat serum for 30 min. Subsequently, the sections were incubated with primary antibody against *α*-SMA, CD31 as well as collagen-III diluted in TBS buffer, overnight at room temperature. After that, the secondary antibody was added dropwise, and the nucleus was counterstained with DAPI, washed with acidified water, and sealed with neutral gum. Finally, the fluorescence image was analyzed.

### 2.5. Western Blotting

The total protein was extracted by lysate, and the protein concentration was detected by a protein concentration detection kit and a microplate reader. Then the protein was added to the loading buffer, heated in boiling water for 10 min, and denatured. Next, the protein samples were treated with 12% SDS-PAGE. After SDS-PAGE, the protein samples were transferred onto the membrane, sealed with 0.5% skim milk for 2 h at room temperature, and incubated with primary antibodies (Abcam) at 4°C. The next day, the protein samples were taken out and incubated with secondary antibodies at room temperature. Finally, the optical density of the target strip was analyzed by the gel image processing system. Primary antibodies purched form abcam, and NOX2, NOX4 (dilution in 1 : 800), p-PI3K, Total-PI3K, p-AKT, Total-AKT, p-P70S6K, Total-P70S6K, HIF-1*α* (dilution in 1 : 1000), and *β*-actin (dilution in 1 : 3000).

### 2.6. Mouse C166 Cell Culture and Lentivirus Infection

The mouse EC line C166 was used as an EC cellular model in our *in vitro* experiment and cultured with the DMEM supplemented with 5% fetal bovine serum and 1% penicillin streptomycin at 37°C and 5% CO_2_ (v/v). The culture medium was replaced 2 to 3 days, and the cells were passaged when the cell adherence area reached 80% of the culture dish. Before lentivirus infection, C166 cells were treated with serum-free medium overnight and infected with lentiviruses (MOI = 10.0) (empty lentivirus in the model group and miR-372-3p KD lentivirus in the miR-372-3p KD group), combined with or without tLY294002, a PI3K inhibitor, treatment. When the cell growth density reached 60%, 1/2 volume of the culture medium containing the corresponding infection complex virus was replaced, at 4 h after infection, the culture medium was supplemented, at 24 h after infection, a new culture medium was replaced, and at 48 h after infection, the infection rate was observed under the fluorescence microscope to determine the infection rate.

### 2.7. Tube Formation Assay of ECs

The concentration of ECs in the logarithmic growth phase was adjusted to 2 × 10^5^ C166 cells/mL, and high-concentration and low-growth-factor Matrigel was added to a precooled 96-well culture plate. The concentration of LY294002 was 5 *μ*M, and the high glucose (HG, 30 mM) concentration was 25.6 mmol/L glucose [31, 32]. After 24 h of incubation, 3 fields of view were randomly selected in each well and photographed (100×). Finally, the differences in the length of the mesh branches and the area of the mesh structure among groups were detected using the ImageJ.

### 2.8. Target mRNA Prediction and Pathway Enrichment Analysis

GSE26887, GSE112556, and GSE146621 datasets were downloaded from the GEO database. The differential analysis between the normal group and DCM group was performed with |LogFC| >1.5 and adjP < 0.01 as the thresholds to obtain the DEGs using the edgeR package in R. In addition, Bayesian method was adopted to analyze differentially expressed miRNAs in the three datasets. To assess the potential target of miR-372-3p, its parental mRNA was obtained using the TargetScan and mirDIP. The function enrichment analysis was carried out according to the GO annotation and the KEGG pathway database using an R-based Bioconductor package data probe.

### 2.9. Immunofluorescence Staining for Collagen-III in Mouse Myocardial Sections

After dewaxed to water by gradient elution, 4*-μ*m-thick mouse myocardial tissue sections were firstly incubated overnight at 4°C using collagen-III primary antibody (diluted at 1: 100). After the sections were washed 3 times (5 min/each) at room temperature and incubated with a secondary antibody at room temperature for 2 h. Lastly, the sections were observed under an optical microscope, and all data were analyzed with Image-Pro 6.0 software.

### 2.10. Q-PCR

Total RNA was isolated by an RNA extraction kit (Solarbio, China) and reverse transcribed into cDNA by PrimeScript RT Master Mix (Takara Bio). qRT-PCR was performed with a SYBR Green system (Takara) according to the following parameters: 95°C for 10 min, followed by 40 cycles of 95°C for 10 s, and 60°C for 50 s. For miRNA expression, U6 were used as internal reference controls for miRNA expression, respectively, and relative expression was calculated using the 2^−*ΔΔ*^Ct method and was used to calculate the relative expression levels of miR-372-3p. Primers: miR-372-3p, forward 5′-TTT CAC GAC GCT GTA AAC TCG CA-3′, reverse 5′ -GTG CAG GGT CCG AGG T-3′; U6, forward 5′-GCT TCG GCA GCA CAT ATA CTA A-3′, reverse 5′-AAC GCT TCA CGA ATT TGC GT-3′.

### 2.11. Statistical Analysis

GraphPad Prism 6.0 software was used to analyze experimental data. Measurement data were expressed as (*x̅*±*s*). The data were compared between two groups from different countries using the *t*-test method and compared among groups using the univariate analysis of variance (ANOVA). *P* < 0.05 represented that the difference was statistically significant. All experiments in this study were conducted independently at least three times.

## 3. Results

### 3.1. Effect of miR-372-3p KD on Cardiac Dysfunction in DCM Mice

To validate the effect of miR-372-3p on cardiac dysfunction in DCM mice, we established miR-372-3p KD mouse models of DCM by STZ injection as described in the “Materials and Methods.” Quantitative ultrasound methods were employed to investigate the effect of miR-372-3p KD on left ventricular function. The results illustrated that LVFS and LVEF declined in DCM mice, indicating that DCM induces conspicuous cardiac dysfunction and systolic dysfunction (Figures 1(a) and 1(b)). The results also revealed that LVFS and LVEF were elevated in the miR-372-3p KD group compared with those in the model group (*P* < 0.05, Figures 1(a) and 1(b)), suggesting that miR-372-3p KD efficiently improves DCM-induced cardiac dysfunction. Furthermore, DCM mice also exhibited a high heart-to-body weight (HW/BW) ratio demonstrating cardiac hypertrophy, which was decreased by miR-372-3p KD. The above findings illustrated that miR-372-3p KD significantly improved left ventricular dysfunction and cardiac hypertrophy in DCM mice, *n* = 7/group.

### 3.2. Effect of miR-372-3p KD on Myocardial Interstitial Fibrosis

Myocardial interstitial fibrosis and hypertrophy are crucial pathophysiological characteristics of DCM. Masson's trichrome staining of mouse myocardial tissues was conducted to evaluate the effect of miR-372-3p KD on cardiac hypertrophy and interstitial fibrosis. As shown in Figure 2(a), the myocardial tissues exhibited significant structural anomalies, excessive fibrosis, and increased collagen fibers in model group. On the contrary, miR-372-3p KD markedly improved these pathological anomalies in myocardial tissues of DCM mice. According to Masson and immunofluorescent analysis results, the ratio of the fibrotic area to the total area as well as fibrotic immunofluorescent intensity in myocardial tissues was increased in the model group compared with that in the miR-372-3p KD group (*P* < 0.05, Figure 2(b)). It could be concluded that miR-372-3p KD improved myocardial interstitial fibrosis and remodeling in DCM mice, *n* = 7/group.

### 3.3. Effect of miR-372-3p KD on Angiogenesis

Angiogenesis is a crucial player in tissue growth and homeostasis. Numerous studies have shown that angiogenesis acts as a positive mediator of pathologic cardiac remodeling in DCM. Immunofluorescence staining was performed to investigate the effect of miR-372-3p KD on angiogenesis in myocardial tissues of mice. As revealed by representative staining images in Figure 3(a), angiogenesis was significantly increased in miR-372-3p KD mice at the tissue level, implying a marked increase in the amount of blood vessels and *α*-SMA-positive tissues in miR-372-3 KD mice. As shown in Figure 3(b), the neovascularization was notably promoted in comparison with that in model group. The above findings suggested that miR-372-3p KD might accelerate cardiac remodeling by increasing angiogenesis in DCM mice, *n* = 7.

### 3.4. Effect of miR-372-3p KD on the AKT/mTOR/HIF-1*α* Pathway

Numerous previous studies have highlighted that the PI3K/AKT/mTOR/p70S6K signaling pathway plays a vital role in the development of neovascularization. Phosphorylation of PI3K, P70S6k, mTOR, AKT, and HIF-1*α* in the myocardial tissues of mice was determined by Western blotting. HIF-1*α* is another crucial downstream protein of mTOR, which plays a vital role in cell proliferation and angiogenesis. The protein and mRNA expression levels of these molecules were compared among the control, model, and miR-372-3p KD groups. The results manifested that the protein and mRNA expressions of p-PI3K, p-P70S6k, p-mTOR, p-AKT, and HIF-1*α* and NADPH oxidase 2 (NOX2) and NOX4 in the miR-372-3p KD group were higher than those in the model and control groups, showing statistically significant differences (Figure 4(a), *P* < 0.01). However, there were no significant differences in the protein and mRNA expressions of these molecules between the control group and the model group (Figure 4(b)). The above findings implied that miR-372-3p is an upstream target of the PI3K/AKT/mTOR/HIF-1*α* signaling pathway, regulating the angiogenesis in DM mice, *n* = 4.

### 3.5. Involvement of the PI3K Signaling Pathway in miR-372-3p KD-Induced Angiogenesis in HG-Stimulated C166 Cells

Next, we determined whether miR-372-3p KD regulates angiogenesis during DM through activating the PI3K signaling pathway in C166 cells. C166 cells were transfected with miR-372-3p KD lentivirus, and then they were stimulated with or without HG medium for 12 h. LY294002, a PI3K inhibitor, was employed in the current study. To further confirm the effect of miR-372-3p KD on the AKT/mTOR/HIF-1*α* signaling pathway, the expressions of p-PI3K, p-AKT, p-mTOR, p-P70S6K, HIF-1*α*, NOX2, and NOX4 in cells were examined by Western blotting. The results exposed that miR-372-3p KD increased the protein and mRNA expressions of p-PI3K, p-AKT, p-mTOR, p-P70S6K, and HIF-1*α*in C166 cells (Figures 5(a) and 5(b), *P* < 0.01), indicating that miR-372-3p KD activates the AKT/mTOR/HIF-1*α* signaling pathway *in vitro*. Moreover, pretreatment with LY294002 markedly diminished this uptrend in the miR-372-3p KD group (Figures 5(a) and 5(b)). Immunofluorescence staining was used to examine the formation of the tubular structure in C166 cells. As shown in Figure 5(c), miR-372-3p KD significantly increased the formation of the tubular structure in C166 cells compared with miR-372-3p NC group (*P* < 0.05). Furthermore, LY294002 weakened the tube formation in the miR-372-3p KD group, *n* = 4. However, the number of tubes formed was not significantly different between the miR-372-3p KD + LY294002 group and the miR-372-3p NC + LY294002 group (*P* > 0.05, Figure 5(c)). The above findings implied that the PI3K signaling pathway is involved in miR-372-3p KD-induced angiogenesis in HG-stimulated C166 cells.

### 3.6. Results of Comprehensive Bioinformatics Analysis of DCM

The putative target of miR-372-3p was identified to explore the molecular mechanisms of miR-372-3p in DCM. TargetScan and mirDIP were employed for the bioinformatics prediction. Among all the potential target genes of miR-372-3p, PIK3CA was selected (Figures 6(a) and 6(b)). DCM-related gene expression profiles were retrieved from GEO datasets (GSE26887, GSE112556, and GSE146621), from which the DEGs were obtained with |Log(FC)| >1.5 and adjP < 0.05 were obtained. Next, heatmaps were plotted to demonstrate the distribution of significant DEGs in GSE26887 and GSE112556. Additionally, PIK3CA was among the downregulated DEGs (Figures 6(c) and 6(d)). Based on the data from GSE146621, a volcano map was plotted to visualize the DEGs, including PIK3CA (Figure 6(e)).

GO enrichment and KEGG pathway enrichment analyses were carried out to investigate the putative function of DEGs in DCM. Most DEGs from GSE26887 and GSE112556 were primarily involved in biological processes, such as angiogenesis, angiogenesis, inflammatory response, nervous system development, patterning of blood vessels, cardiac ventricle morphogenesis, immune system process, protein phosphorylation, cell surface receptor signaling pathway, response to lipopolysaccharide, and negative regulation of Notch signaling pathway (Figures 6(f) and 6(g)). KEGG pathway enrichment analysis for GSE26887 revealed that the DEGs were mainly involved in the PI3K/AKT signaling pathway, HIF-1*α* signaling pathway, NOD-like receptor signaling pathway, and NF-*κ*B signaling pathway (Figure 6(h)). To further investigate the interaction of these DEGs in DCM, the interaction PPI network was built using STRING database according to the data from GSE26887. By using the plug-in CytoHubba in Cytoscape software, PIK3CA was validated as a hub gene and play a crucial role in DCM (Figures 6(j)–6(i)). The above findings indicated that PIK3CA is a potential target of miR-372-3p, and it is a hub gene crucial for DCM.

## 4. Discussion

Wide-range studies have shown that angiogenesis plays a critical role in the progression of DCM [33, 34]. miRNAs, small noncoding RNAs, are referred to as negative posttranscriptional regulators of gene expression by binding to the 3′UTR of large target messenger RNAs (mRNAs) [35]. Various studies have confirmed that miRNAs are beneficial diagnostic and therapeutic markers for controlling DCM [36]. As a crucial member of the miRNA family, miR-372-3p has been described to play a significant role in various diseases [37–39]. However, the specific function of miR-372-3p in DCM remains elusive.

Here, we focused on the potential role and mechanism of miR-372-3p in DCM. Firstly, we established miR-372-3p KD mouse models of DCM by injection of STZ. Quantitative ultrasound results showed that DCM reduced the LVFS and LVEF but increased LVIDd and LVIDs, indicating that it induces apparent cardiac dysfunction and systolic dysfunction. However, LVFS and LVEF were elevated by miR-372-3p KD, suggesting that miR-372-3p KD efficiently improves the DCM-induced cardiac dysfunction. Furthermore, miR-372-3p KD also increased the HW/BW ratio, displaying its role in alleviating DCM-induced hypertension resulting in impaired levels of myocardial blood supply, and cardiac hypertrophy correlates with reduced capillary density and may lead to subsequent myocardial ischemia and HF, and the hypoxic environment-induced angiogenesis improves blood flow and revascularization and suppresses and inhibits the fibrotic progression, thereby fortifying myocardial function and promoting cardiac repair and myocardium survival [40–43]. This study was focused on miR-372-3p effects on the angiogenesis and neovascularization formation and DCM therapy.

It has been previously confirmed that myocardial interstitial fibrosis is a crucial pathophysiological characteristic of DCM [44]. In this study, Masson's trichrome staining and immunofluorescence staining revealed that the myocardial tissues exhibited significant structural anomalies, excessive fibrosis, and increased collagen fibers in model group, but miR-372-3p KD markedly improved these pathological anomalies in myocardial tissues of DCM mice, suggesting that miR-372-3p KD improves myocardial interstitial fibrosis and remodeling in DCM mice. In addition, emerging evidence indicates that hyperglycemia-induced increase in glucose autooxidation, protein glycation, and oxidative degradation of glycated proteins leads to an excessive generation of oxidative stress responses under diabetic conditions, and furthermore, hyperglycemia myocardial metabolism results in ROS overproduction; in conclusion the higher levels of ROS in the heart, the higher the amount of oxidative stress produced, forming a vicious cycle, and furthermore, ROS has been considered the harmful and deleterious effects for heart remodeling and dysfunction in diabetes [24, 26]. In the pathology of DCM, the angiogenesis is a crucial player or cure in tissue growth and homeostasis and acts as a benefit mediator for cardiac remodeling in DCM [45, 46]; previous studies indicated that excessive mitochondrial ROS generation limits angiogenic capacity or causes defective angiogenesis in microvascular endothelial cells [47, 48]; our immunofluorescence staining showed that angiogenesis was significantly enhanced in the miR-372-3p KD group, implying a marked increase in the number of blood vessels. Furthermore, the neovascularization analysis exposed that the number of new blood vessels was markedly increased in the miR-372-3p KD group compared with that in the model group, suggesting that miR-372-3p KD might accelerate cardiac remodeling by increasing angiogenesis in DCM mice. The PI3K/AKT signals are the major promoter for angiogenesis. They are inhibited by oxidative stress, and in turn, they reversely suppress the burst of oxidative stress [49–52]. Remarkably, it has been shown recently that the PI3K/AKT/mTOR/p70S6K signaling pathway plays a vital role in the development of neovascularization [19]. Moreover, HIF-1*α* is another crucial downstream protein of mTOR, which plays a vital role in cell proliferation and angiogenesis [53]. Phosphorylation of PI3K, P70S6k, mTOR, AKT, and HIF-1*α* in myocardial tissues of mice was determined by Western blotting. The results revealed that the protein and mRNA expressions of p-PI3K, p-P70S6k, p-mTOR, p-AKT, and HIF-1*α* in the miR-372-3p KD group were higher than those in the model and control groups, suggesting that miR-372-3p is an upstream target of the PI3K/AKT/mTOR/HIF-1*α* signaling pathway regulating angiogenesis in DCM mice. Furthermore, the oxidative stress could directly destroy the ECs and further inhibits the expression of HIF-1*α*, so the suppression of oxidative stress or the activation of PI3K is the key promoter for neovascularization [19, 37, 38, 51, 54]. Additionally, we determined whether miR-372-3p KD regulates angiogenesis during DM through activating the PI3K signaling pathway in C166 cells. Western blotting results exposed that miR-372-3p KD increased the protein and mRNA expressions of p-PI3K, p-AKT, p-mTOR, p-P70S6K, and HIF-1*α*in C166 cells. Immunofluorescence staining results demonstrated that miR-372-3p KD significantly increased the tubes formed in C166 cells compared with miR-372-3p NC, but this increase was diminished by LY294002. Besides, LY294002 also markedly diminished the increased expression levels of p-PI3K, p-AKT, p-mTOR, p-P70S6K, and HIF-1*α* in the miR-372-3p KD group, suggesting that the PI3K signaling pathway is involved in miR-372-3p KD-induced angiogenesis in HG-stimulated C166 cells.

Furthermore, DCM-related gene expression profiles were retrieved from the GEO datasets (GSE26887, GSE112556, and GSE146621) to obtain DEGs. Heatmaps and volcano map were plotted to screen the DEGs, and it was found that PIK3CA was among the downregulated DEGs. Later, bioinformatics analysis demonstrated that PIK3CA was a potential target of miR-372-3p and a hub gene crucial for DCM. The limitations of this study lie in the deficiency of single-cell transcriptomics as well as cells communicating signals, such as myocardial fibroblasts and inflammatory cells, so such technology should be replenished, and moreover, the cre-loxP mice should be further established to research the further and precise roles of cell subtypes in DCM, and more mechanisms about myocardial remodeling should be carried on under miR-372-3p KD situation, and furthermore, the levels of miR-372-3p may be used as a clinical indicators to predict the DCM' prognosis.

In conclusion, miR-372-3p KD might protect against DCM by accelerating angiogenesis through activating the PI3K/AKT/mTOR/HIF-1*α* signaling pathway or suppressing oxidative stress. Additionally, PIK3CA, a potential target of miR-372-3p, is also a hub gene crucial for DCM. The findings of this study provide a novel evidence for the protective effects of miR-372-3p KD and afford novel potential treatments for patients with DCM.

## Figures and Tables

**Figure 1:** Effect of miR-372-3p KD on cardiac dysfunction. (a) Representative echocardiography in the control, model, and miR-372-3p KD groups. (b) Statistical analysis for LVFS, LVEF, and HW/BW ratio in the control, model, and miR-372-3p KD group. (c) RT-qPCR analysis of relative expression of miR-372-3p. *n* = 7/group, ^∗∗^*P* < 0.05: model group *vs.* miR-372-3p KD group. HW/BW: heart weight/body weight.

**Figure 2:** Effect of miR-372-3p KD on myocardial interstitial fibrosis. (a) Representative images of Masson's trichrome staining of myocardial tissues. Ratio of fibrotic area to total area. Bar: 1.25 mm; (b) the immunofluorescence staining from collagen-III of mouse myocardial tissues. Bar: 50 *μ*M; data were presented as means ± SEM. *n* = 7/group, ^∗∗^*P* < 0.05: model group *vs.* miR-372-3p KD group.

**Figure 3:** Effect of miR-372-3p KD on angiogenesis. (a) Immunofluorescence staining of *α*-SMA and CD31 was performed to examine the neovascularization in myocardial tissue sections. (b) Statistical analysis was performed to show the relative amount of new blood vessels in myocardial tissue sections. Bar: 50 *μ*M; data were presented as means ± SEM. *n* = 7/group, ^∗∗^*P* < 0.01: model group *vs.* miR-372-3p KD group.

**Figure 4:** Effect of miR-372-3p KD on the AKT/mTOR/HIF-1*α* signaling pathway. (a) Protein expressions of p-PI3K, PI3K, p-AKT, AKT, mTOR, p-mTOR, P70S6K, and p-P70S6K HIF-1*α* in the control, model, and miR-372-3p KD groups were identified by Western blotting. *β*-Actin was considered as a loading control. (b) Statistical analysis was performed to examine the expressions of p-PI3K, PI3K, p-AKT, AKT, mTOR, p-mTOR, P70S6K, p-P70S6K, and HIF-1*α* in myocardial tissues. (c) Protein expressions of NOX2 and NOX4 in the control, model, and miR-372-3p KD groups were identified by Western blotting. *β*-Actin was considered as a loading control. (d) Statistical analysis was performed to examine the expressions of NOX2 and NOX4 in myocardial tissues. Data were presented as means ± SEM, *n* = 4/group, ^∗^*P* < 0.05 and ^∗∗^*P* < 0.01: model group *vs.* miR-372-3p KD group.

**Figure 5:** Involvement of the PI3K signaling pathway in miR-372-3p KD-induced angiogenesis in HG-stimulated C166 cells. (a) Protein expressions of p-PI3K, PI3K, p-AKT, AKT, mTOR, p-mTOR, P70S6K, p-P70S6K, and HIF-1*α* in the control, model, and miR-372-3p KD groups treated with or without LY294002. *β*-Actin was considered as a loading control, and the statistical analysis was performed to present the p-PI3K, PI3K, p-AKT, AKT, mTOR, p-mTOR, P70S6K, p-P70S6K, and HIF-1*α* in the control, model, and miR-372-3p KD groups with or without LY294002. (b) Protein expressions of NOX2 and NOX4 in the control, model, and miR-372-3p KD groups treated with or without LY294002. *β*-Actin was considered as a loading control, and the statistical analysis was performed to present the NOX2 and NOX4 in the control, model, and miR-372-3p KD groups with or without LY294002. (c) The number of tubes formed in each group. Data were presented as means ± SEM, Bar: 200 *μ*M, *n* = 4/group, ^∗^*P* < 0.05 and ^∗∗^*P* < 0.01: model group *vs.* miR-372-3p KD group.

**Figure 6:** Comprehensive bioinformatics analysis in DCM. (a) Identification of mRNAs that hypothetically regulated miR-372-3p based on miRDB and TargetScan databases. (b) Target sequences of miR-372-3p in the 3′-UTR of PIK3CA. (c and d) Heatmaps were sketched to illustrate the DEGs in DCM using microarray GSE26887 and GSE112556 datasets. (e) A volcano plot was sketched to illustrate the DEGs in DCM using microarray GSE146621 dataset. (f and g) GO enrichment analysis for biological processes of DEGs using microarray GSE26887 and GSE112556 datasets. *P* < 0.05 denotes significant enrichment. (h) Scatter plot of KEGG enrichment analysis of DEGs using microarray GSE26887 dataset. *P* < 0.05 denotes significant enrichment. (i) The PPI network of DEGs was constructed according to the data from GSE26887. (j) PIK3CA was identified as a hub gene.

## Data Availability

The datasets used and analyzed during the current study are available from the corresponding author on reasonable request.

## Abbreviations

DCM: Diabetic cardiomyopathy
miRNA: microRNA
STZ: Streptozotocin
KD: Knockdown
PI3K: Phosphoinositide 3-kinase
AKT: Protein kinase B
mTOR: Mammalian target of rapamycin
HIF-1*α*: Hypoxia-inducible factor-1*α*
VEGFs: Vascular endothelial growth factors
P70S6K: p70 ribosomal protein S6 kinase
UTRs: 3′ untranslated regions
LVIDd and LVIDs: Left ventricular internal diameter end diastole and end systole
LVFS: Left ventricular fractional shortening
EF: Ejection fraction
*α*-SMA: Alpha-smooth muscle actin
ROS: Reactive oxygen species
NOX: NADPH oxidase
SDS-PAGE: Sodium dodecyl sulfate polyacrylamide gel electrophoresis
EC: Endothelial cell
DMEM: Dulbecco's modified eagle medium
DEGs: Differentially expressed genes
NF-*κ*B: Nuclear factor-kappa B
PPI: Protein-protein interaction.
